# LncRNA NDRG1 aggravates osteosarcoma progression and regulates the PI3K/AKT pathway by sponging miR-96-5p

This article has been retracted.

**DOI:** 10.1186/s12885-022-09833-5

**Published:** 2022-07-04

**Authors:** Zhen Wang, Yanting Wei, Hao Zhu, Lingfeng Yu, Jie Zhu, Qixiu Han, Ziying Liu, Jianhao Huang, Yan Zhu, Gentao Fan, Qikai Tang, Ji Qian, Xi Chen, Guangxin Zhou

**Affiliations:** 1 Department of Orthopaedics, Jinling Hospital, Nanjing Medical University, Zhongshan Road 305, Nanjing, 210002 China; 2 Department of Epidemiology and Biostatistics, School of Public Health, Nanjing Medical University, Tianyuan East Road 818, Nanjing, 211166 China; 3 Department of Orthopaedics, Affiliated Jianhu Hospital of Nantong University, Yancheng, China; 4 Department of Orthopaedics, Jinling Hospital, Nanjing University, Nanjing, China; 5 Department of Orthopaedics, Jinling Hospital, Southern Medical University, Nanjing, China; 6 Department of Neurosurgery, Jiangsu Province Hospital and Nanjing Medical University First Affiliated Hospital, Nanjing, China; 7 Department of Digestion Medicine, Affiliated Yixing Hospital of Jiangsu University, Yixing, China

**Keywords:** Osteosarcoma, LncRNA NDRG1, miR-96-5p, Proliferation, Migration, EMT, PI3K/AKT pathway

## Abstract

**Background:**

Osteosarcoma (OS) is the most common primary malignant bone tumors in children and adolescents. Large numbers of studies have focused on the long non-coding RNA (lncRNA) that plays essential roles in the progression of osteosarcoma. Nevertheless, the functions and underlying mechanisms of LncRNA NDRG1 in osteosarcoma remain unknown.

**Methods:**

Differentially expressed lncRNAs between osteosarcoma and adjacent normal tissues were identified through RNA sequencing. The role of LncRNA NDRG1 in osteosarcoma proliferation and metastasis were investigated through in vitro and in vivo functional experiments. The interaction between LncRNA NDRG1 and miR-96-5p was verified through bioinformatic analysis and luciferase reporter assay. Regulation relationship between LncRNA NDRG1 and miR-96-5p was further evaluated by the rescue experiments. Additionally, the changes in the expression of epithelial-mesenchymal transition (EMT) and the PI3K/AKT pathway were verified by Western blot.

**Results:**

LncRNA NDRG1 was up-regulated in osteosarcoma cell lines and tissues and the expression of LncRNA NDRG1 was correlated with the overall survival of osteosarcoma patients. Functional experiments exhibited that LncRNA NDRG1 aggravated osteosarcoma proliferation and migration in vitro; meanwhile, animals experiments showed that LncRNA NDRG1 promoted osteosarcoma growth and metastasis in vivo. Mechanistically, LncRNA NDRG1 was found to aggravate osteosarcoma progression and regulate the PI3K/AKT pathway by sponging miR-96-5p.

**Conclusions:**

LncRNA NDRG1 aggravates osteosarcoma progression and regulates the PI3K/AKT pathway by sponging miR-96-5p. Therefore, LncRNA NDRG1 could act as a prognostic marker and a therapeutic target for osteosarcoma in the future.

**Supplementary Information:**

The online version contains supplementary material available at 10.1186/s12885-022-09833-5.

## Introduction

Osteosarcoma (OS) is the most common malignant bone tumor which accounts for approximately 56% of bone sarcomas and typically affects children, adolescents and young adults [1, 2]. Such bone tumor is associated with highly aggressive and unfavorable prognoses [3]. Current therapies for osteosarcoma incorporate neoadjuvant chemotherapy, definite surgery and adjuvant chemotherapy [4]. With the advance of the treatment to osteosarcoma, the 5-year survival rate among patients with localized osteosarcoma is approximately 60% but is only 20% among patients with metastases or recurrent disease [5]. Therefore, it is important to clarify the molecular mechanism underlying OS progression so as to provide effective treatment for OS patients in the future [6].

Long non-coding RNAs (lncRNAs) are defined as transcripts of more than 200 nucleotides with no potential of coding protein. Many published articles reveal that lncRNAs play essential roles in the regulation of cell proliferation, migration, invasion, apoptosis, drug resistance and chromatin remodeling [7–10]. Moreover, lncRNAs could act as competing endogenous RNAs (ceRNAs) that sponge microRNAs (miRNAs) to regulate the translation of down-stream messenger RNA (mRNA) [11]. Over the last few years, lncRNAs have gradually been recognized to take part in the progression of OS as well. For example, lncRNA DANCR was recognized as a competitive endogenous RNA which promotes ROCK1-mediated proliferation and metastasis by decoying of miR-335-5p and miR-1972 in osteosarcoma [12]. LncRNA SNHG16 aggravated osteosarcoma progression by acting as the ceRNA of miR-1285-3p [6].

MicroRNAs (miRNAs) are considered as short noncoding RNAs with the length of approximately 23 nucleotides [13]. MiRNAs play important roles in regulating genes expression through directly repressing translation of mRNA. Increasing research revealed that miRNAs are dynamic, exhibiting different expression level in different tissue and diseases, and closely related to the initiation and progression of osteosarcoma [14]. Nowadays, many studies validated that lncRNAs could regulate initiation, proliferation, and metastasis of malignant tumors by sponging miRNAs [15, 16].

In our research, we exhibited a newly screened lncRNA in osteosarcoma: LncRNA NDRG1. By reverse transcription-quantitative PCR (RT-qPCR), we found that LncRNA NDRG1 was up-regulated significantly in osteosarcoma cell lines (MG63, U2OS, HOS and 143B) and tissues, and functional experiments including CCK8, EdU, transwell assay and wound healing assay showed that LncRNA NDRG1 aggravated proliferation and migration of osteosarcoma in vitro. Animal experiments showed that LncRNA NDRG1 promoted OS proliferation and metestasis in vivo. Mechanistically, LncRNA NDRG1 was shown to aggravate osteosarcoma progression and regulate the PI3K/AKT pathway by sponging miR-96-5p. Our study shed lights onto the design of novel therapeutic targets to treat osteosarcoma.

## Materials and methods

### Specimens collection

A total of 18 osteosarcoma patients were included into the study. OS tissues and paired adjacent normal tissues were obtained from Jinling Hospital (Nanjing, China) from January 2018 to January 2020. The study was reviewed and approved by the Ethics Committee of Jinling Hospital (Nanjing, China). And all the patients provided informed written consent authorizing the use of specimens for the intended research. All resected specimens were stored at − 80 °C prior to RNA extraction. Clinical baseline imformation of the patients are presented in Table 1.

**Table 1:** The relationship between clinicopathological features and LncRNA NDRG1 expression in 18 osteosarcoma patients

*p < 0.05, **p < 0.01, chi-square test

### Cell culture

Human OS cell lines (MG63,U2OS, HOS and 143B) and human osteoblast cell line (hFOB 1.19) were obtained from the Cell Bank of the Chinese Academy of Sciences (Shanghai, China). All types of cell were cultured in DMEM (Hyclone; Thermo Fisher Scientific, Inc.) supplemented with 10% fetal bovine serum (FBS) (Gibco; Thermo Fisher Scientific, Inc.), 100 U/ml of penicillin (Life Technologies) and 100 μg/ml streptomycin (Life Technologies) at 37 °C in 5% CO_2_ and 95% air.

### Cell transfection

Three different small interfering (si)RNAs against LncRNA NDRG1 and miR-96-5p mimics, mimics NC, miR-96-5p inhibitor and inhibitor NC were designed and synthesized by Ribobio (Guangzhou, China); LncRNA NDRG1 over-expression plasmid (Lnc-NDRG1) was constructed and synthesized by Genomeditech (Shanghai,China); and transfected into MG63 and 143B cells using Lipofectamine® 3000 (Invitrogen; Thermo Fisher Scientific, Inc.). Cells were collected 48 h after transfection, and the knockdown or over-expression efficiency was detected by reverse transcription-quantitative PCR (RT-qPCR). The lentivirus-containing short hairpin RNA(shRNA) targeting LncRNA NDRG1 was purchased from GenePharma(Shanghai, China), the shRNA was transfected into 143B cell line, after transfecting for 48 h, the cells were selected with puromycin (2 μg/mL) for 2 weeks to construct stable LncRNA NDRG1 knock down cell line. The sequences of LncRNA NDRG1 siRNA, overexpression plasmid and the sequences of miR-96-5p mimics and inhibitor are listed in Tables S1, S2 and S3.

### RNA extraction and RT-qPCR

Total RNA was extracted from the cultured cells and tissues using Trizol Reagent (Invitrogen, CA, USA) according to the manufacturer’s instruction. For the quantification of miRNA, 0.2 μg of total RNA obtained from cultured cells or tissues was reverse-transcribed to cDNA using AMV reverse transcriptase (TaKaRa, Dalian, China), the real-time PCR analyses were performed using SYBR Green dye(Invitrogen) with LightCycler96 System (Roche, IN, USA). For the quantification of lncRNA and mRNA, 1 μg of total RNA was reverse-transcribed to cDNA using Oligo d(T) primer (TaKaRa, Dalian, China), the real-time PCR analyses were performed using SYBR Green dye(Invitrogen) with LightCycler96 System (Roche, IN, USA). All reactions were run in triplicate. After the reactions were complete, the cycle threshold (CT) values were determined with the LightCycler96 software. A comparative CT method was used to compare each condition to the control reactions. In miRNA RT-PCR reaction, U6 was used as an internal control; in lncRNA RT-PCR reaction, GAPDH was used as an internal control, and the relative level was calculated with the eq. 2^−ΔΔCT^. The sequences of the primers used in the present study are listed in Table S4.

### Nucleus and cytoplasm extraction

Nuclear and cytoplasmic fractions were isolated with the reagents in a PARIS™ kit (AM1556, Thermo Fisher Scientific, Waltham, USA). MG63 and 143B cells were lysed in Cell Fraction Buffer on ice for 10 min. Subsequently, after centrifugation at 500 g for 3 min at 4 °C, the supernatant was collected as the cytoplasmic fraction. Then, the pelleted nuclei were washed with Cell Fraction Buffer and used as the nuclear fraction.

### Cell viability assay

The proliferation capability of OS cells (MG63 and 143B) were assessed by cell counting kit-8 assay (CCK-8) according to the manufacturer’s instruction. The transfected cells were seeded into 96-well plates (5 × 10^^3^ cells/well). At 12, 24, 36, 48 and 60 h after transfection, 10 μl of CCK-8 reagent was added to the test well and incubated for 2 h at 37 °C away from light. The absorbance was measured at a wavelength of 450 nm.

### EdU assay

5-Ethynyl-2′-deoxyuridine(EdU) assay was conducted with Cell-LightTM EdU Apollo567 kit (Guangzhou Ruibo Biotechnology). The siRNA or over-expression plasmid of LncRNA NDRG1 or mimics or inhibitor of miR-96-5p were transfected into MG63 and 143B cells. After transfection for 24 hours, MG63 and 143B cells were seeded in 48-well plates(Corning). When the density of cells turned to 80%, reagent A was added to the medium and cells were cultured for another 4 hours. Then, according to the manufacturer’s instruction, the cells were stained. When the staining was done, photos were taken under the microscope (EVOS M7000; Thermo Fisher) at 100 × .

### Wound healing assay

Wound healing assays were performed to evaluate the migration ability of osteosarcoma cells. After transfection for 24 h, MG63 and 143B cells were seeded into six-well plates (8 × 10^^5^ cells/well). After seeding for 48 h, pipette tips (200 μl) were used to scrape a straight scratch in the confluent cell layer and then cultured in serum-free medium. After washing the cells with PBS to remove cellular fragments, each wound was imaged at 0 and 24 h under the microscope (EVOS M7000; Thermo Fisher) at 100×. Cell migration was quantified by measuring the relative wound areas with ImageJ.

### Transwell assay

For the transwell assay, after transfection for 24 h, cells suspended in serum-free DMEM medium were seeded into the upper transwell chamber(Corning). In the lower chamber, DMEM containing 20% FBS was filled in the well. After culturing for 36 hours, the filters were fixed in methanol and stained with 0.1% crystal violet. The upper cells of the filters were gently abraded, and the lower cells migrated across the filters were imaged and counted under the microscope(EVOS M7000; Thermo Fisher) at 100×. The numbers of migrated cells were counted and calculated by ImageJ (NIH).

### Luciferase reporter assay

Wild-type and mutant LncRNA NDRG1 fragments were constructed and inserted into the luciferase reporter plasmid(GenePharma, Shanghai, China). Osteosarcoma cells were seeded in 24-well plates and co-transfected with 0.2 μg of firefly luciferase reporter plasmid, 0.2 μg of β-galactosidase (β-gal) expression plasmid (Ambion), and equal amounts (50 pmol) of miR-96-5p mimics, miR-96-5p inhibitor or the negative control RNAs with Lipofectamine 3000 (Invitrogen). The β-gal plasmid was used as the transfection efficiency control. The cells were assayed using a luciferase assay kit 24 h post-transfection (Promega, Madison, WI, USA).

### Western blot

The total proteins were extracted through radio-immunoprecipitation assay(RIPA) (Beyotime, Shanghai, China) supplemented with PMSF. The extracted protein lysates were separated in 10% SDS-polyacryl-amide gel electrophoresis(SDS-PAGE) and transferred to 0.22 μm PVDF membranes (Millipore, Massachusetts, USA). The membrane was sealed with 5% skim milk and then incubated with primary antibodies at 4 °C overnight. Then the membrane was washed 3 times with 1× TBST for 20 min each. Secondary antibodies were incubated for 1 h at room temperature followed by another 3 times of 10-min wash with 1× TBST. After that, the membrane was incubated with ECL substrate (Thermo Fisher, CA, USA) according to the manufacturer’s instructions and the bands were detected with the SuperSignal West Pico chemiluminescence substrate (Pierce, Thermo Scientific). The protein bands were analyzed with ImageJ. The antibodies we used in the experiments are listed in Table S5.

### Animal experiments

Male BALB/c nude mice (4 weeks old) were purchased from the Model Animal Research Center of Nanjing University (Nanjing, China), and randomly divided into two groups (*n* = 5, respectively). 143B cells transfected with a lentiviral vector sh-LncRNA NDRG1 or sh-NC were subcutaneously injected into armpit of nude mice (1 × 10^7^ cells/mice), respectively. The volume of the tumors was measured every week after implantation. The tumor volume was calculated according to the formula: tumor volume [mm^3^] = (length [mm]) × (width [mm])^2^ × 0.52. The mice were sacrificed after 28 days. The xenograft tumors were excised and weighed. Part of the tumors were used for total RNA extraction, and the remains were fixed in 4% paraformaldehyde for 24 h and then processed for hematoxylin and eosin (H&E) staining as well as immunohistochemical staining for Ki67. For the metastasis assay, 143B cells (1 × 10^^5^) were injected into the tail veins of mice (three mice per group). Lung metastasis was monitored with a Xenogen IVIS Spectrum Imaging System (PerkinElmer, USA). After 8 weeks, the lungs of mice were excised under anaesthesia, and the number of lung metastatic nodules were counted and validated using haematoxylin and eosin (HE)-stained sections by microscopy.

### Immunohistochemistry (IHC)

Immunohistochemistry (IHC) was performed according to the manufacturer’s constructions. After the samples were deparaffinized with xylene and rehydrated with ethanol, the samples were incubated with 3% H_2_O_2_ for 5 min to block endogenous peroxidase activity. Then, antigen retrieval was performed by incubating the samples with sodium citrate buffer (pH 6.0) for 20 min at 95 °C, after which the samples were blocked with 5% normal goat serum for 10 min at 20 °C. Subsequently, the sections were incubated with polyclonal antibodies against Ki67(1:500, Servicebio, Wuhan, China) at 4 °C overnight and then incubated with secondary antibodies(1:200, Servicebio, Wuhan, China). The image were captured by Olympus FSX100 microscope (Olympus,Japan).

### Statistical analysis

All date were expressed as mean ± SD. Statistical analyses were performed using Prism software (GraphPad Software 8), and consisted of analysis of variance followed by Student’s t-test when comparing two experimental groups. One-way ANOVA analysis was used to compare the differences among groups. The correlation between LncRNA NDRG1 expression and clinicopathological variables was calculated by the chi-square test. Overall survival (OS) rates were determined using the Kaplan-Meier method. All experiments were triplicated, and *p* < 0.05 was considered significant.

## Results

### LncRNA NDRG1 is up-expressed in osteosarcoma cell lines and tissues, and is associated with poor prognosis

To identify lncRNAs that are essential to osteosarcoma progression, RNA-seq was performed for 5 pairs of OS and adjacent normal tissues(H1812143). And we presented the results of transcripts which the log_2_fold change> 2.5 with heatmap according to our RNA-seq date (Fig. 1 A). Among these transcripts, we increased our screening requirements with p.adj < 0.5 and basemean> 0.65(S.Figure 1A). With the data from CCLE and Lnc2Cancer(S.Fig. 1B-C), we took the intersection and there were 4 transcripts left in the end(S.Figure 1D). Then we selected LncRNA NDRG1(ENST00000521414) as the targert lncRNA to investigate the biological role of lncRNAs in osteosarcoma. Firstly, we investigated the relative expression of LncRNA NDRG1 in osteosarcoma cell lines and tissues. We found that LncRNA NDRG1 was significantly up-regulated in osteosarcoma cell lines (MG63, U2OS, HOS and 143B) compared with normal control cell line (hFOB) and was significantly up-regulated in osteosarcoma tissues compared with adjacent normal tissues as well (Fig. 1 B, C). Kaplan-Meier analysis demonstrated that high expression of LncRNA NDRG1 were associated with poor prognosis of osteosarcoma patients (Fig. 1 D). After that, the baseline information of 18 osteosarcoma patients have been listed and the high expression of LncRNA NDRG1 was correlated with patients’Enneking stage and distant metastasis (Table 1).

**Fig. 1:** LncRNA NDRG1 expression in OS tissues and cell lines. **A.** The results of transcripts with heatmap which the fold change > 2.5 according to our RNA-seq date(H1812143). **B.** The LncRNA NDRG1 expression in four OS cell lines (MG63, U2OS,HOS and 143B) and normal osteoblast cell (hFOB). **C**. The LncRNA NDRG1 expression in 18 pairs of OS and adjacent normal tissue. **D**. Kaplan-Meier analyses of the overall survival of OS patients with high(*n* = 35) and low(*n* = 46) expression levels of LncRNA NDRG1. *P < 0.05, **P < 0.01, ***P < 0.001. (student’s t test)

### LncRNA NDRG1 aggravates the proliferation, migration and EMT of osteosarcoma cells in vitro

In order to investigate the function of LncRNA NDRG1 in the progression of OS, LncRNA NDRG1 siRNA or negative control were transfected into MG63 and 143B cells. The expression of LncRNA NDRG1 was detected by RT-qPCR after transfection for 48 h. LncRNA NDRG1 siRNA transfection resulted in knocking down of LncRNA NDRG1 significantly in OS cells (Fig. 2 A). Then, the effect of LncRNA NDRG1 on OS proliferation was examined by CCK8 and EdU assay. In MG63 and 143B cell lines, knocking down LncRNA NDRG1 led to decreased cell proliferation ability compared with negative control (NC) transfection group (Fig. 2 B-D). In transwell and wound healing assays, we found that LncRNA NDRG1 knocking down reduced the migration ability of OS cells (Fig. 2 E-H). Epithelial to mesenchymal transition (EMT) plays an important role in cancer progression, especially in cancer metastasis [17]. Many previous articles revealed that EMT participates in osteosarcoma progression as well [18–20]. Therefore, we explored the effect of LncRNA NDRG1 on the EMT of osteosarcoma cells. We detected the expression of EMT-related genes E-cadherin, N-cadherin and Vimentin in MG63 and 143B cells by Western blot. And we found that the expression of E-cadherin in si-LncRNA NDRG1 group was significantly increased compared with si-NC group. In contrast, N-cadherin and Vimentin were decreased, such results suggest that LncRNA NDRG1 could promote EMT in osteosarcoma cells (Fig. 2 I-J). After that, we also constructed the over-expression plasmid of LncRNA NDRG1. After transfecting into the MG63 and 143B for 48 h, the expression of LncRNA NDRG1 was detected and we found LncRNA NDRG1 was significantly up-regulated(S.Figure 2A). Then the proliferaton and migration ability was detected by CCK8, EdU assays and transwell, wound healing assays. The results showed that over-expression of LncRNA NDRG1 in OS cells contributes to enhanced ability of proliferation and migration(S.Figure 2B-H). And the expression of E-cadherin in Lnc-NDRG1 group was significantly decreased compared with vector group while N-cadherin and Vimentin were increased(S.Figure 2I-J). All in all, these data indicated that LncRNA NDRG1 aggravates proliferation, migration and EMT of osteosarcoma cells in vitro.

**Fig. 2:** LncRNA NDRG1 promoted proliferation, migration and EMT of osteosarcoma cells in vitro. **A**. The expression of LncRNA NDRG1 was measured by qRT-PCR in MG63 and 143B cell lines after transfecting LncRNA NDRG1 siRNA. **B**. The growth curves of OS cells were evaluated by CCK-8 assays in MG63 and 143B cells. **C, D**. EdU assays was performed to evaluate OS cells proliferation. The samples were imaged at 100× magnification. Scale bar = 100 μm. **E, F**. Transwell assays were performed to assess the migration ability of OS cells. The samples were imaged at 100× magnification. Scale bar = 100 μm. **G, H**. The wound healing assays were performed to assess the OS cells migration ability. The samples were imaged at 100× magnification. Scale bar = 100 μm. **I, J**. The expression of EMT related genes (E-cadherin, N-cadherin and Vimentin) in MG63/143B cells transfected with si-LncRNA NDRG1 or si-NC. All data are presented as the means ± SD of three independent experiments. *P < 0.05, **P < 0.01, ***P < 0.001. (student’s t test)

### LncRNA NDRG1 functions as a sponge of miR-96-5p

It has already been reported that lncRNAs may act as ceRNAs through binding miRNA to regulate the expression of down-stream genes [21]. So, we conducted the nuclear-cytoplasmic fractionation assay firstly, the results indicated that LncRNA NDRG1 was primarily localized in the cytoplasm of MG63 and 143B cell lines (Fig. 3 A) which means LncRNA NDRG1 may exert functions through ceRNA mechanism. Then, to determine the miRNA which interacts with LncRNA NDRG1, we selected two miRNA target prediction databases (miRcode, miRDB) and identified 6 candidate miRNAs(miR-133a-3p, miR-96-5p, miR-1297, miR-34b-5p, miR-449c-5p, miR-182-5p) that may bind to LncRNA NDRG1 (Fig. 3 B) [22, 23]. After that, we detected the expression of such miRNAs in MG63 and 143B cell lines which transfected with LncRNA NDRG1 siRNA or negative control respectively. The results showed that miRNA-96-5p was significantly up-regulated in LncRNA NDRG1 siRNA group compared with negative control group (Fig. 3 C). Therefore, LncRNA NDRG1 may sponge miRNA-96-5p to exert functions. Finally, we conducted the luciferase reporter assay and the results indicated that miRNA-96-5p binds to LncRNA NDRG1 directly (Fig. 3 D-E). Then, we put our emphasize on miRNA-96-5p. RT-qPCR indicated that miRNA-96-5p was low-expressed in osteosarcoma cell lines and tissues (Fig. 3 F-G).

**Fig. 3:** LncRNA NDRG1 functions as a sponge of miR-96-5p and miR-96-5p is low-expressed in osteosarcoma cells and tissues. **A**. Nuclear-cytoplasmic fractionation assay results indicated that LncRNA NDRG1 was mainly localized in the cytoplasm of OS cells. The GAPDH and U6 genes were used as cytoplasmic and nuclear controls, respectively. **B**. Venn diagram showing the overlap of the target miRNAs of NDRG1 predicted by miRcode and miRDB. **C**. The expression levels of six candidate miRNAs in OS cell lines. U6 was used as internal reference. **D**. Predicted binding sites of miR-96-5p and LncRNA NDRG1. **E**. The luciferase activities of the LncRNA NDRG1 luciferase reporter vector (WT or MUT) in MG63 and 143B cells transfected with miR-96-5p mimics or mimics NC. **F-G**. The expression level of miR-96-5p was measured by qRT- PCR in OS cells and OS tissues. miR-96-5p was down-expressed in OS cells and OS tissues. All data are presented as the means ± SD of three independent experiments. *P < 0.05, **P < 0.01, ***P < 0.001. (student’s t test)

### MiR-96-5p suppresses cell proliferation, migration and EMT in vitro

To investigate the biological function of miR-96-5p, miRNA mimics or inhibitor of miR-96-5p were transfected into MG63 amd 143B cell lines. The expression of miR-96-5p was obviously increased in mimics group, and correspondingly decreased in inhibitor group (Fig. 4 A). The ability of proliferation and migration of MG63 and 143B cells were obviously weakened after overexpression of miR-96-5p, while it was enhanced after miR-96-5p knocking down (Fig. 4 B-I). Then, we explored EMT-related genes expression in MG63 and 143B cells which transfected with miR-96-5p mimics or inhibitor. The results showed that the expression of E-cadherin in MG63 and 143B cells transfected with miR-96-5p mimics was significantly increased compared with the mimics NC group; while the expression of N-cadherin and Vimentin were decreased. The expression of E-cadherin in MG63 and 143B cells transfected with miR-96-5p inhibitor was significantly decreased compared with the inhibitor NC group and the expression of N-cadherin and Vimentin were increased (Fig. 4 J-K). Our results indicated that miR-96-5p acts as the role of tumor supressor in osteosarcoma, which could repress osteosarcoma progression by supressing proliferation, migration and EMT. The results were corresponded to previous research [24, 25].

**Fig. 4:** MiR-96-5p suppresses cell proliferation, migration and EMT in vitro. **A**. The expression level of miR-96-5p was detected in MG63 and 143B cells which transfected with miR-96-5p mimics or inhibitor. **B-I**. The effects of miR-96-5p mimics and inhibitor on cell proliferation and migration ability were assessed by CCK-8, EdU assays and transwell, wound healing assays in MG63 and 143B. The samples were imaged at 100× magnification. Scale bar = 100 μm. **J-K**. The expression of EMT related genes in MG63/143B cells transfected with miR-96-5p mimics or inhibitor. All data are presented as the means ± SD of three independent experiments. *P < 0.05, **P < 0.01, ***P < 0.001. (student’s t test)

### MiR-96-5p reverses the oncogenic effects of LncRNA NDRG1 in osteosarcoma cells

Then, we performed the rescue experiments to illuminate whether LncRNA NDRG1 exerts function by sponging miR-96-5p. MG63 and 143B cells were cotransfected with miR-96-5p inhibitor and LncRNA NDRG1 siRNA. The results indicated that the transfection with miR-96-5p inhibitor significantly promoted the proliferation and migration of MG63 and 143B cell lines, and reversed the suppressive effects which induced by transfecting with LncRNA NDRG1 siRNA in CCK-8, EdU, transwell and wound healing assays (Fig. 5 A-G). The effects of LncRNA NDRG1 in the EMT of osteosarcoma cells were reversed by miR-96-5p as well (Fig. 5 H-I). Our results demonstrated that miR-96-5p reverses the oncogenic effects of LncRNA NDRG1 in osteosarcoma cells.

**Fig. 5:** MiR-96-5p reverses the oncogenic effects of LncRNA NDRG1 in osteosarcoma cells. **A-C**. The function of si-Lnc-NDRG1 in proliferation was reversed by miR-96-5p inhibitor in CCK-8 and EdU assay. **D-G**. The function of si-Lnc-NDRG1 in migration was reversed by miR-96-5p inhibitor in transwell and wound healing assay. **H, I**. The expression of EMT related genes in MG63/143B cells transfected with si-NC + inhibitor NC; si-Lnc-NDRG1 + inhibitor NC; si-NC+ inhibitor or si-Lnc-NDRG1 + inhibitor respectively. All data are presented as the means ± SD of three independent experiments. ns. no significance, *P < 0.05, **P < 0.01, ***P < 0.001. (student’s t test)

### LncRNA NDRG1 aggravates osteosarcoma proliferation and metastasis in vivo

In order to investigate the role of LncRNA NDRG1 in tumor proliferation in vivo, 143B cells were stably transduced with lentivirus sh-LncRNA NDRG1 and lentivirus sh-NC respectively. Then, the cells were subcutaneously injected into the armpit of BALB/c nude mice. Four weeks later, the mice were sacrificed and we found that the expression of LncRNA NDRG1 in sh-LncRNA NDRG1 group was down regulated compared with sh-NC group (Fig. 6 A, B). Tumor mass and volume in the LncRNA NDRG1 knocking down group were significantly decreased compared with the control group (Fig. 6 C, D). In addition, IHC staining revealed decreased Ki-67 expression in LncRNA NDRG1 knockdown group (Fig. 6 E). Furthermore, to determine whether LncRNA NDRG1 could promote OS metastasis in vivo, 143B cells transduced with lentivirus luciferase were injected into the tail veins of male nude mice. The fluorescence intensity in the lung in the sh-LncRNA NDRG1 group were significantly lower than the sh-NC group (Fig. 6 F). Moreover, the number of metastatic nodules in the lung in the sh-LncRNA NDRG1 group was notably reduced than the sh-NC group (Fig. 6 G-I). Such results suggested that LncRNA NDRG1 could aggravate osteosarcoma proliferation and metastasis in vivo.

**Fig. 6:** Knocking down LncRNA NDRG1 could inhibit the growth and metastasis of osteosarcoma in vivo. **A**. 143B cells transfected with a lentiviral vector sh-Lnc-NDRG1 or sh-NC were subcutaneously injected into armpit of nude mice (1 × 10^7^ cells per mice, *n* = 5 each group). **B**. The expression of LncRNA NDRG1 in sh-Lnc-NDRG1 group and sh-NC group. **C, D**. The growth rate and tumor weight obviously decreased in sh-Lnc-NDRG1 group compared with sh-NC group. **E**. HE and IHC staining of xenograft tumors. The expression of Ki67 were analyzed based on IHC staining. The samples were imaged at 400× magnification. Scale bar = 50 μm. **F**. Representative image and analysis of luminescence intensity in tail vein-injected mouse models (*n* = 3 for each group). **G, H**. Representative image and HE staining of metastatic lung nodules. The HE staining samples were imaged at 40× magnification. Scale bar = 100 μm. **I**. The number of lung metastatic nodules in sh-NC and sh-NDRG1 group. All data are presented as the means ± SD, *P < 0.05, **P < 0.01, ***P < 0.001. (student’s t test)

### LncRNA NDRG1/miR-96-5p axis regulates the PI3K/AKT pathway in OS cell lines

To further explore the downstream signal pathways of LncRNA NDRG1/miR-96-5p axis, we firstly predicted the downstream genes of miR-96-5p through Targetscan website [26]. Then we predicted the downstream signal pathways of such genes by KEGG pathway enrichment analysis (Fig. 7 A). It is known that the PI3K/AKT signaling is one of the most frequently dysregulated signaling pathways observed in cancer that plays crucial roles in tumor initiation, progression and therapy responses [27]. So we selected the PI3K/AKT signal pathway for further study conbined with our KEGG analysis results. After that, we detected the expression of the genes in the PI3K/AKT pathway by Western blot. And we found that the expression of phosphorylated PI3K (p-PI3K) and phosphorylated AKT(p-AKT) were down-regulated obviously in si-LncRNA NDRG1 group compared with si-NC group while the expression of PI3K and AKT did not exhibit significant difference (Fig. 7 B, C). Then, we explored such genes expression in MG63 and 143B cells which transfected with miR-96-5p mimics or inhibitor. We found that the expression of p-PI3K and p-AKT in MG63 and 143B cells transfected with miR-96-5p mimics was significantly down-regulated compared with the mimics NC group; the expression of p-PI3K and p-AKT in MG63 and 143B cells transfected with miR-96-5p inhibitor was significantly up-regulated compared with the inhibitor NC group. No significant differences in the expression of PI3K and AKT were seen (Fig. 7 D, E). Finally, the effects of LncRNA NDRG1 in the PI3K/AKT pathway of osteosarcoma cells were reversed by miR-96-5p through resecue experiments (Fig. 7 F-G). After that, to detect whether LncRNA NDRG1 exerts function through the PI3K/AKT pathway, rescue experiments among LncRNA NDRG1 and PI3K/AKT pathway were performed. MG63 and 143B cells transfected with LncRNA NDRG1 overexpression plasmid were treated with PI3K inhibitor wortmannin. CCK8 and transwell assays showed that the proliferation and migration ability of OS cells were decreased in wortmannin treated group compared with LncRNA NDRG1 overexpression plasmid tranfected group(S.Figure 3A-D).

**Fig. 7:** LncRNA NDRG1/miR-96-5p axis regulates the PI3K/AKT pathway in OS cell lines. **A**. KEGG pathway analysis of the target genes of miR-96-5p predicted by Targetscan. **B, C**. The relative expression of p-PI3K/PI3K and p-AKT/AKT in MG63/143B cells transfected with si-Lnc-NDRG1 or si-NC. **D, E**. The relative protein expression of p-PI3K/PI3K and p-AKT/AKT in MG63/143B cells transfected with miR-96-5p mimics or inhibitor. **F, G**. The relative protein expression of p-PI3K/PI3K and p-AKT/AKT in MG63/143B cells transfected with si-NC + inhibitor NC; si-Lnc-NDRG1 + inhibitor NC; si-NC+ inhibitor or si-Lnc-NDRG1 + inhibitor respectively. All data are presented as the means ± SD of three independent experiments. ns. no significance, *P < 0.05, **P < 0.01, ***P < 0.001. (student’s t test)

## Disscussion

Nowadays, large number of lncRNAs have been discovered and more evidence indicates that lncRNAs play important roles in the development and progression of multiple cancers [28–30]. As to osteosarcoma, there are many published articles demonstrating that lncRNAs participate in the development of OS by regulating cell proliferation, migration, metastasis, apoptosis and chemoresistance [6, 7, 18, 31, 32]. For instance, LncRNA MALAT1 promotes tumor angiogenesis by regulating microRNA-150-5p/VEGFA signaling in osteosarcoma [33]; LncRNA SNHG16 promotes epithelial-mesenchymal transition by upregulating ITGA6 through miR-488 inhibition in osteosarcoma [34]; LncRNA HCG18 promotes osteosarcoma growth by enhanced aerobic glycolysis via the miR-365a-3p/PGK1 axis [35] and so on.

In this article, we selected LncRNA NDRG1 which has not been reported in osteosarcoma for further study from our own RNA-seq results(H1812143). We proved that LncRNA NDRG1 was up-regulated obviously in osteosarcoma cell lines and tissues. So we supposed that LncRNA NDRG1 may play an important role in the progression of osteosarcoma. To verify our thought, we knocked down or over-expressed LncRNA NDRG1 via siRNA or overexpression plasmid; then the proliferation, migration and EMT abilities were examined. The results exhibited that knocking down LncRNA NDRG1 leads to low proliferation, migration and EMT activity and overexpressing LncRNA NDRG1 leads to high proliferation, migration and EMT activity in both MG63 and 143B cell lines. Moreover, animal experiments demonstrated that LncRNA NDRG1 could aggravate proliferation and metastasis of osteosarcoma in vivo. Such results revealed that LncRNA NDRG1 may take part in the development of osteosarcoma and could be a potential therapeutic target in the future.

Previous studies have proved that the possible mechanisms of lncRNAs was closely associated with the distribution in cells [36]. So we conducted the nuclear-cytoplasmic fractionation assay, the results indicated that LncRNA NDRG1 was primarily localized in the cytoplasm of MG63 and 143B cell lines, which indicated that our lncRNA might function as a miRNA sponge(ceRNA). Therefore, we predicted the down-stream miRNAs through miRNA target prediction databases and confirmed the binding sites between LncRNA NDRG1 and miR-96-5p via the luciferase assay. Our results suggested that LncRNA NDRG1 may exert functions by sponging miR-96-5p. Nevertheless, the function of miR-96-5p in osteosarcoma remains uncertain. Previous studies have demonstrated that miR-96-5p repressed breast cancer proliferation and invasion through Wnt/β-catenin signaling via targeting CTNND1 [37]; miR-96-5p regulated TGF-β/SMAD signaling pathway and suppressed endometrial cell viability and migration via targeting TGFBR1 [38]. Our study indicated that miR-96-5p was significantly decreased in OS cell lines and tissues. Functional experiments demonstrated that miR-96-5p could inhibit OS cell proliferation, migration and EMT in vitro. The results implied that miR-96-5p may play a tumor supressor role in osteosarcoma which were consistent with previous study [25].

Overall, our study first demonstrated the novel LncRNA NDRG1 in osteosarcoma. LncRNA NDRG1 aggravated OS progression and regulated the PI3K/AKT pathway by sponging miR-96-5p. These results validated the interaction between LncRNA NDRG1 and miR-96-5p, such interaction could be a novel pathway in osteosarcoma which could provide a promising therapeutic target for the treatment of OS patients in the future. By the way, miRNA generally pairs to mRNA to regulate the transcription of target genes, and it is a limitation that the we did not study the target gene regulated by miR-96-5p, and we plan to conduct the related research in the future.

## Conclusion

In summary, LncRNA NDRG1 could act as the ceRNA of miR-96-5p, thus aggravated the progression of osteosarcoma and regulated the PI3K/AKT pathway. Therefore, LncRNA NDRG1 may serve as a prognostic marker and a therapeutic target for osteosarcoma in the future.

## Supplementary Information

**Additional file 1: Table S1.** The sequences of Lnc NDRG1 siRNA. **Table S2.** The sequences of Lnc NDRG1 overexpression plasmid. **Table S3.** The sequences of miR-96-5p mimics and inhibitor. **Table S4.** The sequences of the primers used in the present study. **Table S5.** The antibodies we used in the experiments.

**Additional file 2: S.Figure 1.** LncRNA NDRG1 was selected from the intersection. **A.** Transcripts with the log_2_fold change > 2.5; p.adj < 0.5 and basemean> 0.65. **B.** The expression of transcripts in 4 OS cell lines(SJSA, U2OS, Saos2 and MG63) from the CCLE database. **C.** The Venn diagram showed the intersection among RNA-sequence, CCLE and Lnc2Cancer. **D.** Four lncRNAs were left from the intersection

**Additional file 3: S.Figure 2.** LncRNA NDRG1 promoted proliferation, migration and EMT of osteosarcoma cells in vitro. **A**. The expression of LncRNA NDRG1 was measured by qRT-PCR in MG63 and 143B cell lines after transfecting LncRNA NDRG1 overexpression plasmid. **B**. The growth curves of OS cells were evaluated by CCK-8 assays in MG63 and 143B cells. **C-D**. EdU assays was performed to evaluate OS cells proliferation. The samples were imaged at 100× magnification. Scale bar = 100 μm. **E-F**. Transwell assays were performed to assess the migration ability of OS cells. The samples were imaged at 100× magnification. Scale bar = 100 μm. **G-H**. The wound healing assays were performed to assess the OS cells migration ability. The samples were imaged at 100× magnification. Scale bar = 100 μm. **I-J**. The expression of EMT related genes (E-cadherin, N-cadherin and Vimentin) in MG63/143B cells transfected with vector or Lnc-NDRG1. All data are presented as the means ± SD of three independent experiments. *P < 0.05, **P < 0.01, ***P < 0.001. (student’s t test)

**Additional file 4: S.Figure 3.** The function of LncRNA NDRG1 was supressed by wortmannin. **A-B.** The effect of wortmannin on the proliferation of OS cells which transfected with LncRNA NDRG1 overexpression plasmid was detected through CCK8 assay. **C-D.** The effect of wortmannin on the migration of OS cells which transfected with LncRNA NDRG1 overexpression plasmid was detected through transwell assay. The samples were imaged at 100× magnification. Scale bar = 100 μm. All data are presented as the means ± SD of three independent experiments. *P < 0.05, **P < 0.01, ***P < 0.001. (student’s t test)

## Data Availability

The datasets generated and/or analyzed during the current study are available in the GEO repository (https://www.ncbi.nlm.nih.gov/gds/), CCLE database (https://sites.broadinstitute.org/ccle) and Lnc2Cancer database (http://www.bio-bigdata.net/lnc2cancer/).

## Abbreviations

LncRNA: Long non-coding RNA
NDRG1: N-myc downstream regulated 1
OS: Osteosarcoma
miRNA: microRNA
RT-Qpcr: reverse transcription quantitative polymerase chain reaction
EMT: epithelial-to-mesenchymal transition
ceRNA: competing endogenous RNA
CCK8: Cell Counting Kit-8
EdU: 5-Ethynyl-2′-deoxyuridine
GAPDH: Glyceraldehyde-3-phosphate dehydrogenase
shRNA: Short hairpin RNA
IHC: Immunohistochemistry
PI3K: Phosphoinositide 3-kinase
p-PI3K: Phosphorylated phosphoinositide 3-kinase
AKT: α-Serine/threonine-protein kinase
p-AKT: Phosphorylated α-serine/threonine-protein kinase
